The article "Efficacy of Letrozole Combined with Urinary Gonadotropin for Ovulation Induction in Endocrine Abnormal Infertility Patients: A Retrospective Single-Center, Case-Control Study" was retracted in 2023. Reasons: unreliable results or conclusions; lack of ethics approval or compliance; missing or withdrawn patient consent; concerns about the data.

# Efficacy of Letrozole Combined with Urinary Gonadotropin for Ovulation Induction in Endocrine Abnormal Infertility Patients: A Retrospective Single-Center, Case-Control Study

**DOI:** 10.1155/2022/5363754

**Published:** 2022-07-11

**Authors:** Hao Peng, Ben Yuan, Junbiao Mao, Junling Wang, Shuhong Luo

**Affiliations:** ^1^Department of Obstetrics and Gynecology, Huangshi Central Hospital, Affiliated Hospital of Hubei Polytechnic University, Edong Healthcare Group, Huangshi, 435000 Hubei Province, China; ^2^Department of Reproductive Medicine, Huangshi Central Hospital, Affiliated Hospital of Hubei Polytechnic University, Edong Healthcare Group, Huangshi, 435000 Hubei Province, China; ^3^Hubei Province Key Laboratory of Occupational Hazard Identification and Control, Wuhan University of Science and Technology, Wuhan, 430000 Hubei Province, China

## Abstract

**Aims:**

To ask lots of questions and try to find the truth about the medicine-based effectiveness of letrozole (LE) combined with human menopausal gonadotropin (HMG) in the treatment of inability to have children crops patients with endocrine (things that are different from what is usually expected and the effect on ovulation-related chemicals produced by the body).

**Materials and Methods:**

A total of 160 unable to have children crops patients with endocrine things that are different from what is usually expected who were treated in our hospital from March 2019 to March 2022 were selected as the subjects of this look at how things were in the past study and were divided into instance of watching, making a statement group was treated with human menopausal gonadotropin on the basis of the control group. The differences in serum related to the process of making children, chemical produced by the body levels, ovarian function, and ovulation induction effect between the two groups were watched and compared.

**Results:**

After treatment, LH, FSH, PRL, and E_2_ in the observation group were better than those in the control group. The ovarian volume, follicle size, follicle diameter, and endometrial thickness of the two groups of patients were significantly improved, and the observation group was better than the control group. Significance is *P* < 0.05. After treatment, the ovarian volume, follicle size, follicle diameter, and endometrial thickness in the two groups were significantly improved, and the observation group was better than the control group, and the difference was statistically significant (*P* < 0.05). The ovulation rate, pregnancy rate, singleton pregnancy rate, and multiple pregnancy rate of the observation group were higher than those of the control group, and the difference was statistically significant by the chi-square test (*P* < 0.05).

The article "Efficacy of Letrozole Combined with Urinary Gonadotropin for Ovulation Induction in Endocrine Abnormal Infertility Patients: A Retrospective Single-Center, Case-Control Study" was retracted in 2023. Reasons: unreliable results or conclusions; lack of ethics approval or compliance; missing or withdrawn patient consent; concerns about the data.

**Conclusion:**

Letrozole can promote the improvement of sex hormones in infertile patients. After being combined with human menopausal gonadotropin treatment, the follicle development and ovulation of patients are significantly improved, and infertility is improved to a certain extent. It has a certain reference value in the clinical treatment of endocrine abnormal infertility.

## 1. Introduction

There are many reasons for infertility, the most common are tubal blockage, endometriosis, and endocrine abnormalities. However, endocrine abnormalities account for about 60% of female anovulatory infertility, and women's health and pregnancy are seriously affected [1, 2]. For the treatment of endocrine abnormal infertility, early and timely prevention of miscarriage, ovulation induction, and enhancement of luteal function should be treated. However, in recent years, there have been many clinical treatment drugs for endocrine abnormal infertility, but the effect is still not satisfactory, so how to find new drug treatment ideas and drugs are particularly important [3]. Letrozole (LE) is another ovulation induction drug that has attracted more and more attention. Letrozole is a third-generation aromatase inhibitor. A large number of clinical studies have found that it can promote the growth of follicles, and gradually, it is used for ovulation induction therapy in infertile patients with ovulatory disorders [4]. Urinary gonadotropin (HMG) is a commonly used drug for ovulation induction in patients with endocrine abnormal infertility. In recent years, many academic studies have found that urinary gonadotropin can prevent autoimmune diseases, antitumor, and improve lung function and other effects [5, 6]. Based on this, we study that HMG is mainly used for oral administration of LE to promote follicular growth that is not obvious, and when there is no dominant follicle growth, but at this time antral follicles have undergone the initial recruitment of follicles, and intramuscular injection of HMG can effectively reduce the development of multiple follicles and reduce ovarian hyperstimulation syndrome and the incidence of multiple pregnancies. Therefore, the main purpose of our research is to explore more effective ovulation-stimulating drugs and ovulation-stimulating programs, so as to solve fertility problems for patients with endocrine abnormal infertility.

## 2. Material and Methods

### 2.1. Research Object

A total of 160 infertile patients with endocrine abnormalities who were treated in our hospital from March 2019 to March 2022 were selected as the subjects of this retrospective study and were divided into an observation group and a control group with 80 cases in each group according to different treatment methods. Diagnostic criteria are according to the “Clinical Guidelines developed by the American Society of Endocrinology Based on Expert Consensus” [7]. Diagnostic criteria: the patient is 22 to 39 years old, has a normal sexual life after marriage, has not been pregnant for at least 1 year, and has a uterine shape revealed by salpingography. Normal, at least one fallopian tube is unobstructed; the man's semen is routinely normal or slightly less. Pregnancy diagnosis: urine HCG or blood HCG positive 2 weeks after follicular ovulation is detected by ultrasound monitoring, and the positive patient will undergo transabdominal vaginal ultrasound 2 weeks later, and the gestational sac and fetal heartbeat are monitored as clinical pregnancy bit pregnancy.

The article "Efficacy of Letrozole Combined with Urinary Gonadotropin for Ovulation Induction in Endocrine Abnormal Infertility Patients: A Retrospective Single-Center, Case-Control Study" was retracted in 2023. Reasons: unreliable results or conclusions; lack of ethics approval or compliance; missing or withdrawn patient consent; concerns about the data.

### 2.2. Inclusion and Exclusion Criteria

Inclusion criteria: (i) 3 blood was collected on days 2~5 of the menstrual cycle to detect serum prolactin, follicle-stimulating hormone (FSH), luteinizing hormone (LH), estradiol (E), and testosterone (T). The diagnosis of anovulation was confirmed by blood sampling for progesterone on the 21st to 23rd day of the menstrual cycle; (ii) all patients were monitored by vaginal ultrasound for anovulation in natural cycles before treatment according to those who had normal sexual intercourse without contraception for 1 year without pregnancy; (iii) all patients were confirmed by tubal iodine oil imaging for patency of at least one side of the fallopian tube and normal semen analysis of the husband.

Exclusion criteria: (i) in patients with genetic disorders, patients with psychiatric abnormalities, patients aged >38 years, patients with combined other nonendocrine disorders; (ii) other causes of infertility, patients with previous history of infectious diseases, patients allergic to our study drugs, patients with combined uterine fibroids or uterine malformations; (iii) patients allergic to our study drugs, and patients with combined uterine fibroids or uterine malformations.

### 2.3. Methods

In the control group, letrozole was used; LE 2.5 mg was administered orally twice a day for 5 d starting from the 5th day of the menstrual cycle or the 5th day of withdrawal bleeding, and transvaginal B-mode vaginal ultrasound was performed on the 11th-12th day of the menstrual cycle to observe the follicles and endometrial growth. 10,000 U was injected to induce LH peak and promote ovulation, and intercourse was instructed within 24-36 hours after the injection. 48 hours later, transvaginal B-mode vaginal ultrasound was performed to observe whether the follicles ruptured. In the observation group, human menopausal gonadotropin was administered orally on day 5 of menstrual cycle or day 5 of withdrawal bleeding, LE 2.5 mg twice daily for 5 d. Transvaginal B-mode ultrasound was performed on days 11-12 of menstrual cycle to monitor follicle size and endometrial thickness, and HMG75 was given to those without dominant follicles (follicle diameter < 14 mm). In the absence of dominant follicles (follicle diameter < 14 mm), HMG 75 IU was given once every other day by intramuscular injection. When there is a mature follicle (follicle diameter greater than or equal to 18 mm), HCG 6000-10000 U will be injected intramuscularly to induce LH peak and ovulation. After 48 hours of HCG injection, a transvaginal B-echo examination was performed and those with follicular rupture were given oral progesterone capsules (Kinect) 100-200 mg daily or dydrogesterone (Dafeton) 10 mg daily for 14 days for luteal support. 14 days later, urine HCG or blood HCG was checked to determine if pregnancy was present. If pregnancy was confirmed, a transabdominal B-ultrasound examination was performed 2 weeks later, and clinical pregnancy was determined if an intrauterine gestational sac and fetal heartbeat were seen on ultrasound (including ectopic pregnancy). All infertile patients will experience withdrawal bleeding after discontinuation of progesterone and will be treated with the next cycle if this ovulation cycle fails. During the monitoring process, if the endometrium is thin, the patient will be treated with 14 g of oral Glivec daily, oral aspirin 100 mg daily, and prednisone 7.5 mg daily to improve the endometrial blood circulation, thus improving the tolerance of the endometrium and reducing the body's immune rejection of the fertilized egg, which will play a negative immune regulating role to facilitate the fertilized egg's implantation.

The article "Efficacy of Letrozole Combined with Urinary Gonadotropin for Ovulation Induction in Endocrine Abnormal Infertility Patients: A Retrospective Single-Center, Case-Control Study" was retracted in 2023. Reasons: unreliable results or conclusions; lack of ethics approval or compliance; missing or withdrawn patient consent; concerns about the data.

### 2.4. Statistical Analysis

Repeated measure analysis of variance between groups was used to measure the measurement expressed as mean ± standard deviation (*X* ± SD). Material. Count data expressed as a percentage (%) were tested by *χ*^2^. Univariate and logistic multivariate regression analysis was used to compare the influencing factors, and the risk factors with significant differences were screened. Correlation test using logistic regression linear correlation analysis. Included data that did not conform to a normal distribution were described by M (QR), using the Mann-Whitney test. All statistical tests were two-sided probability tests. The statistical significance was *P* < 0.05.

## 3. Results

### 3.1. Comparison of General Data

The comparison of general data such as mean age, body mass index, duration of infertility, and type of disease between the two groups was not statistically significantly different by the *t*-test and chi-square test (*P* > 0.05). See Table 1.

### 3.2. Serum Sex Hormone Comparison

Before treatment, there was no significant difference in serum sex hormones between the two groups (*P* > 0.05); after treatment, the FSH, PRL, and E_2_ of the observation group were lower than those of the control group, but the LH of the observation group was higher than that of the control group. The difference was significant (*P* < 0.05). See Table 2 and Figure 1.

### 3.3. Comparative Ovarian Function

After treatment, ovarian (total space occupied by something), hair root size, hair root (distance or line from one edge of something, through its center, to the other edge), and (related to the uterus) thickness improved very much in both groups and were better in the (instance of watching, noticing, or making a statement) group than in the comparison group, and this difference was a big change in numbers that means something important (*P* < 0.05). See Table 3 and Figure 2.

### 3.4. Ovulation Promotion Effect

The ovulation rate, pregnancy rate, singleton pregnancy rate, and multiple pregnancy rate of patients in the observation group were higher than those in the comparison group, and the difference was statistically significant by the chi-square test (*P* < 0.05). See Figure 3.

## 4. Discussion

Endocrine abnormal infertility is a major problem for women of reproductive age seeking fertility, and exploring different ovulation promotion protocols to solve the infertility problem in patients with endocrine abnormal infertility is the main aim of our study [8]. The main feature of endocrine abnormal infertility is sporadic ovulation or anovulation, and the mechanism of normal follicular growth and development is the process of follicles developing autonomously from the initiating follicle to the antral follicle and finally to the mature follicle [9]. It undergoes four stages of initial recruitment, autonomous growth, regulated growth, differentiation, and final maturation, during which it undergoes two recruitments, initial recruitment and cyclic recruitment [10]. Patients with endocrine abnormal infertility have significantly more follicles in the initial recruitment stage compared to the normal population, while their follicles' further development of cyclic recruitment is inhibited; therefore, during ovulation promotion in patients with endocrine abnormal infertility, too small a dose of ovulatory drugs leads to increased recruitment of small follicles in the ovary [11]. Without dominant follicle formation, excessive doses are prone to the simultaneous development of multiple follicles once the threshold is exceeded, leading to multiple pregnancies [12]. Letrozole decreases estrogen levels by inhibiting aromatase in the body, thus relieving the negative feedback inhibition of estrogen on the hypothalamus and pituitary gland and secreting FSH, which promotes follicle development and ovulation [13]. In addition, it blocks the conversion of androgens to estrogens, causing androgens to accumulate in the ovaries, increasing follicle sensitivity to follicle-stimulating hormone (FS), causing follicle growth, and promoting ovulation [14]. Letrozole drug has a short half-life, it does not consume estrogen receptors, and FSH released from the pituitary gland does not continue to rise and does not lead to multiple follicle growth, which can lead to ovulation of a single dominant follicle [15]. HMG has strong pharmacological effects and is prone to complications such as multiple pregnancies, our study was mainly used when oral letrozole promotes follicle growth is not obvious, and there is no dominant follicle growth [16]. Sinus follicles experiencing initial follicular recruitment in the early follicular phase followed by intramuscular HMG can effectively reduce the development of multiple follicles and also reduce the HMG dosage and the occurrence of multiple pregnancies [17]. HMG can be applied alone with a starting dose of 75 U per day as a minimum dose, and HMG can also be combined with letrozole or clomiphene to increase the sensitivity of the ovary to HMG and also reduce the HMG dosage [18].

The article "Efficacy of Letrozole Combined with Urinary Gonadotropin for Ovulation Induction in Endocrine Abnormal Infertility Patients: A Retrospective Single-Center, Case-Control Study" was retracted in 2023. Reasons: unreliable results or conclusions; lack of ethics approval or compliance; missing or withdrawn patient consent; concerns about the data.

FSH, PRL, and E_2_ were lower in the observation group than those in the comparison group after treatment in our study; however, LH was higher in patients in the observation group than in the comparison group, suggesting that letrozole combined with urotropin can promote the improvement of sex hormones in infertile patients. The reason may be that reproductive hormones such as LH, FSH, and E_2_ have important roles in ovulation and conception [19]. LH and FSH are both secreted by the anterior pituitary gland, and both can synergistically stimulate follicle development, maturation, and discharge and can promote sex hormone production and secretion [20]. E_2_ is secreted by the follicles in the ovaries, and this hormone can promote increased endometrial thickness and provide conditions for conception [21]. LH, SH, and E_2_ levels are too low, then the sinus follicles are recruited and selected, inhibiting the formation of dominant follicles and leading to the occurrence of anovulation [22]. The combination of letrozole with urotropin significantly increases reproductive hormone levels and facilitates the production of estrogen in the late follicular development and postovulatory luteal phase, which acts on the endometrium and increases its thickness, making it more conducive to pregnancy [23]. In addition, the short half-life of letrozole is associated with the disappearance of the drug's effect of reducing estrogen levels in the late follicular development, thus reducing the effect on endometrial proliferation and avoiding the occurrence of multiple pregnancies and early abortions [24].

The article "Efficacy of Letrozole Combined with Urinary Gonadotropin for Ovulation Induction in Endocrine Abnormal Infertility Patients: A Retrospective Single-Center, Case-Control Study" was retracted in 2023. Reasons: unreliable results or conclusions; lack of ethics approval or compliance; missing or withdrawn patient consent; concerns about the data.

In our study, ovarian volume, follicle size, follicle diameter, and endometrial thickness improved significantly in both groups after treatment and were better in the observation group than in the comparison group, indicating that letrozole combined with urotropin improves ovarian function. The reason is that the application of clomiphene or letrozole in the early follicular phase can recruit follicles, and the combination with urotropin can reduce the large number of follicle initiation caused by the use of urotropin alone [25], reducing the dominant follicle on the one hand, while decreasing the dose of this drug. Letrozole in combination with urotropin promotes ovulation and eliminates ovulatory disturbances in patients [26]. The reason may be that letrozole combined with urotropin addresses the low intrinsic follicle-stimulating hormone in patients, maintains the expected growth rate of follicles, promotes follicle development and maturation, and increases ovulation rate [27]. The mechanism of LE ovulation promotion may be achieved through central and peripheral mechanisms [28]. Centrally, it prevents estrogen synthesis in early menstruation by inhibiting aromatase activity, decreasing estrogen levels in the body, relieving negative feedback inhibition of the hypothalamus/pituitary gland, prompting increased endogenous Gn secretion, and stimulating follicle development [29]. In the periphery, by binding to the ferrous heme atoms of the aromatase complex and competing with endogenous substrates to bind the active site of aromatase, the conversion of androgens to estrogens is blocked in the ovary due to LE, leading to a temporary increase in androgens [30].

There are some limitations in our study: first, the samples selected were from our hospital, inclusion-exclusion were subjective and small, and there may be regional differences in the study results; second, a parallel, double-blind design was not used, or it may lead to biased results. Finally, the trend of clinical treatment effects over a long follow-up period was not studied in depth. As mentioned above, letrozole can promote the improvement of sex hormones in infertile patients, and the follicular development and ovulation of patients were significantly improved after the combined addition of urotropin treatment, which improved infertility to some extent and has a certain reference value in the clinical treatment of endocrine abnormal infertility.

The article "Efficacy of Letrozole Combined with Urinary Gonadotropin for Ovulation Induction in Endocrine Abnormal Infertility Patients: A Retrospective Single-Center, Case-Control Study" was retracted in 2023. Reasons: unreliable results or conclusions; lack of ethics approval or compliance; missing or withdrawn patient consent; concerns about the data.

## Figures and Tables

**Figure 1:** Comparison of serum sex hormones (all the comparisons of serum sex) (chemicals produced by the body): data in this study were entered into excel software by the first author and the similar author (match up each pair of items in order), and the independent samples *t*-test was performed as the mean Â ± standard moving away. The results showed that after treatment, the FSH (b), PRL (c), and E_2_ (d) of the (instance of watching, noticing, or making a statement) group were lower than those of the control group, but the LH (a) of the (instance of watching, noticing, or making a statement) group was higher than that of the control group, and the difference was a big change in numbers that means something important (*P* < 0.05).

**Figure 2:** Comparative ovarian function (all serving to compare two or more things): ovarian function data in this study were entered into excel software by the first author and the similar author (match up each pair of items in order), and the independent samples *t*-test was performed using the mean *Â* ± standard moving away. The results showed that after treatment, the ovarian (total space occupied by something), hair root size, hair root (distance or line from one edge of something, through its center, to the other edge), and (related to the uterus) thickness of the two groups of patients were very much improved, and the (instance of watching, noticing, or making a statement) group was better than the control group, and the difference was a big change in numbers that means something important (*P* < 0.05).

**Figure 3:** Effectiveness of ovulation promotion: all effectiveness of ovulation promotion data in this study were entered into excel software by the first author and the corresponding author, respectively, and the mean ± standard deviation was used to carry out the independent samples *t*-test. The results showed that the ovulation rate, pregnancy rate, singleton pregnancy rate, and multiple pregnancy rate of the observation group were higher than those of the control group, and the difference was statistically significant by the chi-square test (*P* < 0.05).

**Table 1:** Comparison of general data (*n*, ($\overset{¯}{x}\pm s$)).

Group	Average age (years)	Body mass index (kg/m^2^)	Duration of infertility (years)	Disease type		
				Amenorrhea lactation syndrome	Hypoestrogenemia	Kallmann syndrome
Comparison group (80)	26.78 ± 5.32	24.78 ± 3.09	2.31 ± 0.67	40	23	17
Observation group (80)	26.62 ± 5.66	24.62 ± 3.10	2.29 ± 0.95	42	22	16
*χ* ^2^/*t*	0.130	0.231	0.131	0.100	0.031	0.038
*P*	0.897	0.818	0.913	0.752	0.860	0.845

The article "Efficacy of Letrozole Combined with Urinary Gonadotropin for Ovulation Induction in Endocrine Abnormal Infertility Patients: A Retrospective Single-Center, Case-Control Study" was retracted in 2023. Reasons: unreliable results or conclusions; lack of ethics approval or compliance; missing or withdrawn patient consent; concerns about the data.

**Table 2:** Analysis of sex hormones in two groups of patients ($\overset{¯}{x}\pm s$).

Group comparison group (80)	LH (miv/mL)		FSH (miv/mL)		PRL (ng/mL)		E_2_ (pg/mL)	
	Before therapy	After treatment	Before therapy	After treatment	Before therapy	After treatment	Before therapy	After treatment
Observation group (80)	19.44 ± 3.23	76.27 ± 10.14	8.34 ± 1.25	12.81 ± 2.82	57.23 ± 10.57	22.67 ± 3.24	64.76 ± 7.15	194.45 ± 9.15
Group	19.80 ± 3.22	70.37 ± 10.20	8.31 ± 1.64	14.27 ± 2.81	57.24 ± 6.53	18.23 ± 2.26	64.75 ± 7.26	185.57 ± 9.16
*t*	-0.706	3.669	0.130	-3.280	0.007	10.053	0.009	6.135
*P*	0.481	≤0.001	0.897	≤0.001	0.994	≤0.001	0.993	≤0.001

**Table 3:** Comparison of ovulation therapy and ovarian function between the two groups ($\overset{¯}{x}\pm s$).

Group	Ovarian volume (ml)	Follicle size (cm)	Follicle diameter (cm)	Endometrial thickness (cm)
Comparison group (80)	4.98 ± 1.10	0.41 ± 0.10	1.41 ± 0.17	7.71 ± 1.56
Observation group (80)	4.10 ± 1.08	0.74 ± 0.11	1.63 ± 0.15	9.50 ± 1.82
*t*	5.106	-19.855	-8.679	-6.679
*P*	≤0.001	≤0.001	≤0.001	≤0.001

## Data Availability

No data were used to support this study.
